# Investigation on the Differences in the Failure Processes of the Cortical Bone under Different Loading Conditions

**DOI:** 10.1155/2022/3406984

**Published:** 2022-11-17

**Authors:** Xiaofeng Dai, Ruoxun Fan, Huajie Wu, Zhengbin Jia

**Affiliations:** ^1^Department of Traffic Engineering, Yangzhou Polytechnic Institute, Yangzhou 225127, China; ^2^Department of Aerospace Engineering, Jilin Institute of Chemical Technology, Jilin 132022, China; ^3^Department of Mechanical and Aerospace Engineering, Jilin University, Changchun 130025, China

## Abstract

Cortical bone is a transversely isotropic material, and the mechanical properties may be related to the loading direction on the osteon. Therefore, analyzing the differences in the failure processes of cortical bone under different loading conditions is necessary to explore the measures for reducing the incidence of fracture. In this study, to investigate the effects of different loading directions on the fracture performance in the cortical bone, a numerical method that could simultaneously simulate the failure processes in the cortical bone structure under compression and bending loads was established based on continuum damage mechanics theory. The prediction accuracy and feasibility of the numerical method were first verified by comparing with the corresponding experimental results. Then, the differences in the failure process and fracture performance of the same cortical bone structure under compression and bending loads were investigated. The simulation results indicated that for the same structure, the slip-open failure mode appeared under compression load, and the crack propagated along a certain angle to the loading direction; the tension-open failure mode appeared under bending load, and the crack propagated along the direction perpendicular to the loading direction. Meanwhile, the fracture load was greater and the fracture time was later in the compression than in the bending condition. These phenomena stated that discrepant failure processes and fracture patterns occurred in the same cortical bone structure under different loading conditions. The main reason may be related to the tension–compression asymmetry and transversely isotropic characteristics in the cortical bone material. The fracture simulations in the cortical bone under different loading conditions could improve the prediction accuracy in bone biomechanics and provide the prevention method for cortical bone damage and fracture.

## 1. Introduction

Predicting and observing the failure process in cortical bone are necessary to explore the measures for reducing the incidence of fracture [1]. The fracture simulation in cortical bone mainly includes two processes [2, 3]. The first step is element damage in the cortical bone finite element (FE) model, which may cause crack initiation; then, the increasing number of damage elements may lead to crack propagation with loading, and the elastic modulus in the damage element gradually decreases until the element fails. When the failed element reaches a certain percentage or the crack propagates to a certain location, a complete fracture occurs [4].

Bone fracture simulation based on continuum damage mechanics (CDM) theory first conducts a gradual decrease in element stiffness until the element fails and then simulates the complete failure when the failed element reaches a certain degree, which is similar to the actual failure process in the cortical bone [5, 6]. Thus, many studies accurately simulated the cortical bone fracture using the numerical method with CDM theory. Hambli et al. predicted the failure process in the human proximal femur coupled with a quasi-brittle damage law to describe the initiation and progressive propagation of multiple cracks [7, 8]. Soni et al. investigated the parametric uncertainties on the fracture behavior of the proximal femur [9]. Fan et al. predicted the critical failure strain for the cortical bone structure [10]. All the above studies used the numerical method with CDM theory to explore the fracture performance of the cortical bone under compression load. Furthermore, Dapaah et al. simulated the fracture process in the bovine cortical bone structure during three-point bending load, and the prediction accuracy in the simulations with CDM theory was verified by comparing with the experimental data [11, 12]. Giner et al. also used the same method to predict the critical energy release rate of the bovine cortical bone under three-point bending load [13].

These studies concluded that the fracture model based on CDM theory could accurately simulate the failure process in cortical bone, and the complete fracture caused by compression or bending loads had been particularly discussed. However, cortical bone material expresses tension–compression asymmetry and transversely isotropic characteristics [14, 15]. The fracture performance under different loading conditions may be discrepant, and the material properties may be related to the loading direction on the osteon [16]. Current fracture simulations mainly forced on the unidirectional loading, and few investigated the differences in the failure processes in the cortical bone under different loads. Thus, the effects of different loading directions on the fracture process and performance of cortical bone structure were not clear.

Therefore, to investigate the effects of different loading directions on the fracture performance in cortical bone, a numerical method based on CDM theory that could simultaneously simulate the failure processes in the cortical bone structure under compression and bending loads was established in this paper. Cortical bone specimens were first obtained from rat femurs. The rat femoral cortical bone FE models were established based on the microimage of the femur specimens, and the compression and three-point bending experiments on the rat femurs were performed. Then, the compression and three-point bending fracture simulations for the corresponding cortical bone structures were conducted, and the accuracy of the fracture simulation was verified by comparing with the experimental results. Finally, the differences in the failure processes and fracture mechanical properties of the same cortical bone structure under compression and bending loads were investigated. The fracture simulation for the same cortical bone under different loading conditions could help improve the prediction accuracy in bone biomechanics and explore the prevention methods for bone damage and fracture.

## 2. Materials and Methods

### 2.1. Description of the Compression and Three-Point Bending Experiments

Eight right femurs were obtained from eight healthy 3-month-old Wister rats, and the soft and muscle tissues attached to the femur were all removed. Four right femurs were cut along the femoral axis to obtain a 5 mm cortical bone as the compression test specimen, and another four intact femurs were directly used as the three-point bending test specimens.

The compression experiment was performed by placing the four cortical bone specimens vertically on the electronic testing machine, and the compression speed was set to 0.5 mm/min to implement quasi-static load. The preload of 30 N was performed before the test to ensure the specimens would not slide during the compression test [17]. Four intact femur specimens were placed transversely on the electronic testing machine in turn to perform the three-point bending test. The compression span was set to 20 mm, and the indenter of the testing machine was driven down at a uniform speed of 0.5 mm/min until complete failure [18].

### 2.2. Establishment of the Cortical Bone Finite Element Model

Based on the micro-CT scan on the femur specimens, the microimages of the femur were obtained by SKYSCAN software, and then the images were imported into MIMICS software to reconstruct the geometric model of the rat femur, and the cortical bone FE model in the middle femur and the intact femur FE model were established by ABAQUS software applying C3D4 element [19].

Rigid circular plates were established above and below the cortical bone to simulate the boundary condition in the compression experiment. Frictionless interactions were set among the upper and lower rigid plates and the cortical bone models. All the degrees of freedom in the lower rigid plate were constrained, and axial compression displacement was applied to the upper rigid plate, as shown in Figure 1(a). A rigid indenter and two rigid braces were established above and below the femur model to simulate the boundary condition in the three-point bending experiment. The locations among the rigid indenter, braces, and the femur model were the same with the experiment. Because the loading location was on the cortical bone in the middle of the femur, the trabecular bone was not created in the femur FE model to reduce computing cost. Frictionless interaction was set between the upper rigid indenter and the femur model, and the TIE interactions were set between the lower braces and the femur model [20]. All the degrees of freedom in the lower rigid braces were constrained, and the axial displacement was applied to the upper rigid indenter, as shown in Figure 1(b).

### 2.3. Fracture Simulation on the Cortical Bone Finite Element Model

This study simulated the cortical bone fracture based on CDM theory. The stress–strain relationship after the onset of the damage can be expressed as [5, 21]:

(1) $$\begin{array}{c} \sigma_{ij}=\left(1-D\right)C_{ijkl}\varepsilon_{kl}, \end{array}$$

where **σ**_ij_ is the stress tensor in the element, *D* is the damage variable in the element, **C**_ijkl_ is the elasticity tensor of the undamaged material, and *ε*_kl_ is the strain tensor in the element.

The damage variable expression in the cortical bone material was [4, 21]:

(2) $$\begin{array}{c} \begin{array}{l} D=0\left(\varepsilon_{pri}\leq \varepsilon_{y}\right);D=0.95*\left|\varepsilon_{pri}\right|\left(\varepsilon_{y}<\varepsilon_{pri}<\varepsilon_{f}\right);\\ D=0.95\left(\varepsilon_{pri}\geq \varepsilon_{f}\right), \end{array} \end{array}$$

where *ε*_pri_ is the maximum or minimum principal strain in the element, *ε*_y_ is the critical yield strain in the cortical bone material, and *ε*_f_ is the critical failure strain in the cortical bone material.

In the simulation, the positive and negative values of the principal strain in the element in the FE model should be judged first to determine the damage in tension or compression. Then, the UMAT subroutine automatically compared the maximum or minimum principal strain with the critical tensile or compressive strain in the material to complete the change in the mechanical state of the element. At the initial stage of loading, the cortical bone FE model was in the elastic stage, and no element damage occurred. The principal strain in the element reached the critical yield strain in the cortical bone material with loading, where the maximum principal strain was compared with the critical tensile yield strain and the minimum principal strain was compared with the critical compressive yield strain. The element was gradually damaged and the crack was initiated at the yielding stage. The element stiffness decreased with the increasing damage variable *D*, resulting in the declining apparent stiffness and load-carrying capacity in the cortical bone structure. When the principal strain exceeded the critical failure strain of cortical bone material, where the maximum principal strain was compared with the critical tensile failure strain and the minimum principal strain was compared with the critical compressive failure strain, the element failed. The elastic modulus in the failed element dropped to 5% of the initial value, and lost its bearing capacity. When the failed element accumulated to a certain degree, complete failure occurred on the cortical bone FE model [22]. This provided a complete description of the failure process in the cortical bone FE model based on CDM theory, and this process was implemented by subroutine UMAT in ABAQUS software.

### 2.4. Determination of the Material Parameters in the Finite Element Model

Cortical bone is a transversely isotropic material and expresses asymmetrical mechanical properties in tension and compression [23, 24]. To improve the simulation accuracy, the longitudinal and transverse elastic moduli in the cortical bone FE model were assigned, and the specific values were measured by previous nanoindentation experiment on the femoral cortical bone of 3-month-old Wister rats [25]. The critical yield and failure strain in tension and compression in the cortical bone material needed to be assigned in the UMAT subroutine to perform fracture simulation. The critical failure strain in the femoral cortical bone of the 3-month-old rat has been measured by our previous research, whereas the critical yield strain was not yet known [4, 10]. Therefore, the critical yield strain in the cortical bone material can be obtained by the back-calculation fitting from the experimental data. All the material parameters in the cortical bone FE models could be seen in Table 1.

## 3. Results

### 3.1. Mesh Sensitivity Analysis

Mesh sensitivity analysis was performed to determine the suitable element size for the two types of cortical bone FE model in this paper. Five sizes (30, 40, 50, 60, and 70 *μ*m) were selected to establish the two cortical bone FE models. As shown in Figure 2(a), the predicted fracture load increased with the coarse mesh in the compression condition. When the element size was larger than 60 *μ*m, the fracture load increased violently, which may result in misalignment. Then, as shown in Figure 2(b), the shapes of the load–displacement curves predicted by the cortical bone FE models with different element sizes did not differ much in the three-point bending condition. However, the predicted fracture load and fracture time were slightly advanced with the fine mesh, which indicate that the decrease in the element size may cause an increase in the structural softening rate. Meanwhile, the computational convergence in the cortical bone FE model with the fine mesh was relatively more complete, indicating that the coarse mesh was not conducive to computational convergence. Because the fracture simulation method adopted in this study cannot make the crack through the element, fine element was needed. Considering the computational cost, the element size in the cortical bone FE models established in this paper was all set to 40 *μ*m.

### 3.2. Calibration of the Critical Yield Strain in the Cortical Bone Material

Most of the material parameters in the cortical bone FE model in this paper have been obtained from previous studies, except for the critical yield strain in the cortical bone material. Therefore, back-calculated calibration between the predicted and experimental load–displacement curves was performed to acquire the critical yield strain. Different critical yield strains were repeatedly substituted in UMAT subroutine to conduct fracture simulation until the predicted curves were consistent with the experimental curves for all the cortical bone FE models. The calibration results showed that the critical tensile yield strain was 1.67%, and the critical compressive yield strain was 3.05% in the rat femoral cortical bone.

### 3.3. Comparison of the Fracture Patterns in the Experiments and Simulations

Figure 3(a) shows the damage and failure process of the cortical bone FE model under compression load. Initially, several damage elements appeared on the upper and lower surfaces of the FE model. Then, the main crack was initiated in the lower and middle locations of the FE model, and propagated at an angle to the loading direction from the top and bottom until it penetrated the cortical bone structure, resulting in a complete fracture. The accuracy of the simulated fracture pattern can be compared with the experimental failure picture.  Figure 3(b) shows the damage and failure process of the cortical bone FE model under the three-point bending load. The damage element and crack first appeared on the inferior side of the femur, that was, away from the indenter. As bending increased, the crack began to cross the femoral axis and gradually propagated to the compressive region of the femur until it penetrated the whole femoral section, leading to a complete fracture. Because the loading position set in the simulation was based on the experimental bounding condition, the simulated fracture position was consistent with the experiment.

### 3.4. Comparison of the Experimental and Predicted Load–Displacement Curves

Figure 4 exhibits the predicted load–displacement curves from the compression and bending conditions and the experimental curves. The shapes of the curves obtained from the experiments and fracture simulations were similar. Meanwhile, the differences in the fracture mechanical parameters between the simulations and experiments were not apparent, which indicate the accuracy of the fracture simulation. However, the predicted apparent elastic modulus differed slightly from the experimental results. This may because the elastic modulus assigned to the FE model was the average value of the elastic moduli measured by the nanoindentation experiments, which led to a certain discrepancy between the actual and assigned elastic modulus. The fracture load was greater under compression load than under bending load, and the fracture time was later during compression than during bending. This finding indicated the variances in the fracture mechanical properties existed for the same cortical bone structure under different loading conditions.

## 4. Discussion

In this paper, a numerical method was established to simulate the failure processes of rat femoral cortical bone under compression and three-point bending loads. Then, the reasons for the variances in the fracture performance of the same cortical bone structure under different loads were revealed by observing and analyzing the fracture patterns and fracture mechanical parameters in the simulations and experiments.

The simulation results (Figure 3) first exhibited that different fracture patterns occurred in the same cortical bone structure under compression and bending loads. The slip-open failure mode appeared in the compression condition. The main crack is first produced in the middle, and then propagated along a certain angle to the loading direction. Because the compressive loading direction was vertical and similar to the orientation of the osteon, the oblique crack in the structure should be caused by the combined action of the compressive and shear stresses. Therefore, the compression and shear failures leading to slip-open mode appeared in the cortical bone structure under compression load, which was consistent with the fracture pattern in the compression condition reported in the literature and the corresponding experimental data in this study [22]. The tension-open failure mode appeared on the same cortical bone structure under three-point bending load. Because the crack was produced in the middle of the structure and propagated along the direction perpendicular to the bending load, the fracture was mainly caused by the action of tensile stress, which led to tension-open mode. Several studies also considered that the crack was primarily initiated in the tensile region away from the indenter during the three-point bending experiment on the femur and then gradually propagated to the compressive region of the femur until complete failure occurred [26, 27]. Thus, the tension failure appeared in the cortical bone under bending load, which was similar to the reports in the literature and the corresponding experimental data in this study. These comparisons illustrated the accuracy of the fracture simulation in this paper. Furthermore, the comparison between different simulations also indicated different fracture patterns appeared on the same cortical bone under compression and bending loading conditions. Different fracture patterns would inevitably lead to dissimilar fracture mechanical properties on one structure [28]. The comparison of the load–displacement curves also exhibited that the fracture mechanical parameters of the same cortical bone structure were different under compression and bending loads. That was, the complete failure occurred earlier and the fracture load was lower in the cortical bone structure under bending condition, compared with compression condition.

The variances in the failure processes and fracture performance in the same structure under different loading conditions may be related to the specific material properties in the cortical bone. The cortical bone is a transversely isotropic material [23, 24]. The indenter acted on the transverse structure in the cortical bone during three-point bending while loaded on the longitudinal bone unit during compression. Therefore, the growth in the element strain on the cortical bone structure during compression was faster than that under bending load at the same time. Meanwhile, both the critical compressive yield and failure strain of the cortical bone material were greater than the corresponding critical tensile yield and failure strain due to the asymmetric mechanical properties in tension and compression, so the element in the FE model suffered compressive damage and failure needed for greater principal strain compared with tension condition. Therefore, at the macroscopic level, the fracture load as well as fracture time in the cortical bone structure under compression load was greater and later, which was consistent with the conclusions of the previous study [29].

In calibrating the critical yield strain of the cortical bone material, the calibration strain base was different because of the dissimilar fracture patterns under the two types of loading condition. The main reason for the cortical bone fracture under compression was excessive compression strain, so the critical compressive yield strain was calibrated in the compression condition. The tension failure occurred under bending load, so the critical tensile yield strain was calibrated in the bending condition. This analysis explained why the critical yield strain values calibrated for the same material varied under different loading conditions. Moreover, the ratio of the calibrated critical tensile to compressive yield strain was about 0.55, which was consistent with the previous conclusions, namely, the ratio of the tensile to compressive yield strain in the cortical bone at the tissue level was about 0.6 [30].

The comparisons of the load–displacement curves and fracture patterns between experiments and simulations verified the accuracy and feasibility of the fracture model based on CDM theory. However, inconsistent exponent in the damage variable expression was chosen compared with the references. *D* = 0.95∗|*ε*_pri_|^1^ and the exponent was set to 1 in this paper, and the exponent was set to 2 in most references [5, 7, 9]. The discrepancy in the exponent in the damage variable expression may lead to differences in the decreasing rate of the elastic modulus in the element during the damage and failure processes. The reason for the difference in the settings here was mainly due to the different analysis objects. The fracture model established in the literature mainly focused on trabecular bone structure, whereas this simulation applied to cortical bone structure. The yielding phase in the trabecular bone is more pronounced and longer than that of cortical bone, so the elastic modulus decreases more slowly in the yielding phase during fracture simulation. Considering the shorter yielding phase in the cortical bone structure, the exponent in the damage variable expression was set to 1 to achieve a faster decrease in the elastic modulus of the element. Furthermore, different exponents were applied to perform fracture simulation to investigate the effects of different damage variable expressions on the fracture performance in the paper. Four sets of data with exponents of 1, 1.5, 2, and 3 were used for fracture simulation, and the results showed that the effects of different exponents on the fracture mechanical parameters were almost nonexistent. Therefore, the change in the exponent had no effect on the simulation result because the yielding phase in the cortical bone is not obvious and even the possibility of quasi-brittle fracture. The discrepancy in the exponent in the damage variable expression is a major difference between the cortical bone and trabecular bone in fracture simulation based on CDM theory [31, 32].

Although the fracture processes of cortical bone structures under compression and bending loads can be simulated, certain limitations also existed in this paper. First, the simulation method cannot reflect the effects of different strain rates on the fracture performance of the cortical bone. Different loading speeds have a large effect on the mechanical properties of the cortical bone because most fractures are caused by impact load. The UMAT subroutine prepared in this paper is mainly used to simulate quasi-static loading condition, and the VUMAT subroutine needs to be prepared for impact load, which is also the focus of subsequent research field. Second, due to the limitation of experimental specimens, only four specimens were analyzed and tested for each load, which influenced the calibration of the mean value of cortical bone material parameters. However, the main purpose of this paper was to verify the accuracy of the established fracture simulation method and investigate the differences in the fracture mechanical properties of cortical bone under different loading conditions, so the number of specimens did not have much influence on the simulation results.

## 5. Conclusions

This paper established a numerical method that could simultaneously simulate the failure processes in the cortical bone structure under compression and bending loads based on CDM theory. The comparisons of the load–displacement curves and fracture patterns between the experiments and simulations verified the accuracy and feasibility of the fracture method. Both the experimental and simulated results expressed evident differences in the failure processes of the same cortical bone structure under compression and bending loads. The slip-open failure mode appeared under compression load, and the crack propagated along a certain angle to the loading direction; the tension-open failure mode appeared under bending load, and the crack propagated along the direction perpendicular to the bending load. Meanwhile, the fracture load was greater and the fracture time was later in the compression load than in the bending load. The reason for the differences may relate to the asymmetry in tension–compression and the transversely isotropic characteristics in the cortical bone material. Human cortical bone is always subjected to loads from different directions. The findings in the study stated that load-bearing capacity in each direction was different in cortical bone. Therefore, Clarifying the failure process and comparing the fracture performance of cortical bone in different loading directions may provide preventative measures for different types of cortical bone fractures and theoretical basis for the development of rehabilitation devices in the future.

## Figures and Tables

**Figure 1:** Schematic diagrams of the experiments and simulations on the rat femurs: (a) compression experiment and simulation; (b) three-point bending experiment and simulation.

**Figure 2:** Mesh sensitivity analysis for the femoral cortical bone finite element models: (a) simulation in the compression condition; (b) simulation in the three-point bending condition.

**Figure 3:** Comparison of the fracture patterns between the simulations and experiments: (a) the failure process in the compression simulation; (b) the failure process in the three-point bending simulation.

**Figure 4:** Comparison of the load–displacement curves obtained by the fracture simulations and the experiments: (a) comparison of the predicted and experimental load–displacement curves under compression; (b) comparison of the predicted and experimental load–displacement curves under bending.

**Table 1:** The material parameters in the cortical bone finite element model.

Material parameter	Value	Source
Transverse elastic modulus	30270 MPa	Previous experiment [25]
Longitudinal elastic modulus	32470 MPa	Previous experiment [25]
Poisson's ratio	0.3	References [1, 2]
Critical yield strain in compression	3.05%	Calibration
Critical failure strain in compression	4.35%	Previous conclusion [4]
Critical yield strain in tension	1.67%	Calibration
Critical failure strain in tension	2.61%	Previous conclusion [4]

## Data Availability

The data used to support the findings of this study are available from the corresponding author upon request.

## Abbreviations

FE: Finite element
CDM: Continuum damage mechanics
UMAT: User material.
